The article "Optimal Household Water Access Fosters the Attainment of Minimum Dietary Diversity among Children Aged 6–23 Months in Malawi" was retracted in 2021. Reasons: plagiarism; overlap with other authors' work.

# Optimal Household Water Access Fosters the Attainment of Minimum Dietary Diversity among Children Aged 6–23 Months in Malawi

**DOI:** 10.3390/nu13010178

**Published:** 2021-01-08

**Authors:** Zizwani Brian Chilinda, Mark L. Wahlqvist, Meei-Shyuan Lee, Yi-Chen Huang

**Affiliations:** 1 Graduate Institute of Public Health, China Medical University, 91 Hsueh-Shih Road, North District, Taichung City 40402, Taiwan; bryanchilinda@yahoo.co.uk; 2 Department of Nutrition, China Medical University, 91 Hsueh-Shih Road, North District, Taichung City 40402, Taiwan; mark.wahlqvist@gmail.com; 3 School of Public Health, National Defense Medical Center, No. 161, Section 6, Minquan East Road, Neihu District, Taipei City 11490, Taiwan; mmsl@ndmctsgh.edu.tw; 4 Institute of Population Health Sciences, National Health Research Institutes, 35 Keyan Road, Zhunan, Miaoli County 35053, Taiwan; 5 Monash Asia Institute, Monash University, 5th Floor, H Building, 900 Dandenong Road, Caulfield East, Melbourne, VIC 3145, Australia

**Keywords:** dietary diversity, infants, Malawi, undernutrition, water access, young children

## Abstract

Along with sanitation and hygiene, water is a well-known driver of child undernutrition. However, a more direct role of household (HH) water access in shaping dietary diversity remains unexplored. We assessed the association between HH water access and achievement of minimum dietary diversity (MDD) among young children. We utilized nationally-representative cross-sectional data from the 2015/16 Malawi Demographic and Health Survey, which included 4727 mother–child dyads, respectively, (26.8 ± 6.8 years, range 15–49 years) and (13.9 ± 4.9 months, range 6–23 months). HH water access was categorized as (1) basic or no access, (2) intermediate, or (3) optimal. MDD was defined as feeding a child, during the previous day, at least four of the food groups defined by the World Health Organization. Only 27.7% of the children achieved MDD standards; most of the children who achieved MDD were from HHs with optimal water access (58.4%, *p* < 0.001). However, only 5.9% of the mother–child dyads were from HHs with optimal water access. After adjusting for covariates, children from HHs with optimal water access had higher odds of achieving MDD than those from HHs with basic or no water access (aOR = 1.74, CI = 1.24–2.46). Our results highlight the need to incorporate water-based strategies into national nutritional policies to increase dietary diversity among Malawian infants and young children.

## 1. Introduction

In many countries, less than one-fourth of children aged 6–23 months meet the criteria for dietary diversity and feeding frequency [1]. This stage is the critical window of opportunity to prevent childhood malnutrition. It is a period of growth faltering and malnutrition, since children need more energy and nutrient-dense foods to grow and develop [2,3,4]. Inappropriate complementary feeding practices have been linked to poor dietary diversity and increased risk of undernutrition, illness, and mortality among children under the age of two years [5,6].

The article "Optimal Household Water Access Fosters the Attainment of Minimum Dietary Diversity among Children Aged 6–23 Months in Malawi" was retracted in 2021. Reasons: plagiarism; overlap with other authors' work.

Identifying the factors associated with inappropriate child-feeding behaviors is crucial for designing and implementing effective nutrition interventions, as well as for informing policies. Access to adequate and safe water has been found to affect child nutrition and health outcomes, mainly through water, sanitation, and hygiene (WASH) pathways [7,8,9]. Independent of the WASH pathways, the literature has highlighted three ways in which water might directly impact a child’s dietary diversity. First, water availability affects household food diversity through food choices. People in water-rich regions have higher opportunities to diversify their crops because they can easily grow a wider variety of foods than their counterparts in water-stressed regions [10]. Greater local water availability also increases households’ likelihood of having water-based animal foods such as fish in their diet [11], thus increasing their dietary diversity. Second, water access may also affect dietary diversity by straining household budgets, forcing resource-constrained households to choose between buying water, food, or fuel. In such instances, buying water leaves them with inadequate finances for acquiring an adequate and diverse diet [7,12,13]. Third, water access may affect a child’s dietary diversity through the household food/preparation pathway [14]. Mothers have reported an increased demand for water, during the first 1000 days of a child’s life, for preparing complementary foods and breastfeeding [12]. In a recent cross-country study conducted in 19 sites across 16 low- and middle-income countries, most women cited insufficient water for preparing complementary foods as the main reason for feeding their infants less-preferred foods [15]. Efforts to improve water access to marginalized communities would, thus, be in line with the agendas of the United Nations’ Sustainable Development Goals 2, 3, and 6, which seek to achieve zero hunger and end malnutrition in all its forms, ensure health and well-being for all, and ensure access to water and sanitation for all by the year 2030, respectively [16].

Malawi has one of the highest numbers of undernourished children in sub-Saharan Africa. Approximately 37% of children under five years of age in Malawi are stunted, an indicator of chronic undernutrition that reflects a failure to receive adequate nutrition over a long period [17]. Data from the Malawi Millennium Development Goals (MDG) Endline Survey, 2014 also showed that only 27% of Malawian children aged 6–23 months achieved minimum dietary diversity (MDD) [18]. A child’s chances of attaining MDD also varied across Malawi’s three main geographical regions; the northern and southern regions performed marginally better in this regard than the central region [18]. A similar trend was reported for child stunting rates [17].

The article "Optimal Household Water Access Fosters the Attainment of Minimum Dietary Diversity among Children Aged 6–23 Months in Malawi" was retracted in 2021. Reasons: plagiarism; overlap with other authors' work.

Around 5.6 million people do not have access to safe water sources in Malawi, and poor WASH practices have contributed to about 3000 deaths of children under five years of age, every year [19]. The country has water resources covering 21 percent of its territory, including Lake Malawi, the third largest freshwater lake in Africa. However, high year-on-year population growth rates, increasing demands on its water resources, and lack of infrastructure combine to make Malawi a water-stressed country. This is especially true in rural areas where only 10 percent of people have access to a piped water source [20]. These spatial differences in water availability present an opportunity for exploring the role that household water availability and access, in a broader concept, might play in shaping children’s dietary diversity in Malawi.

In Malawi, a more direct effect of water on infant and young child nutrition remains under- if not unexplored. Against this backdrop, we set out to assess the effect of household water access on MDD standards among Malawian infants and young children, using Demographic and Health Survey (DHS) data. We hypothesized that household water access is positively associated with a child’s achievement of MDD.

## 2. Materials and Methods

### 2.1. Population and Study Design

The data were obtained from the 2015/16 Malawi DHS (MDHS), a survey that provides comprehensive information on childcare, child feeding practices, and relevant sociodemographic information on the household. The data were gathered by trained data collectors and field supervisors using pretested and structured questionnaires. The original questionnaires were in English and were translated into the local Chichewa and Tumbuka languages by highly skilled and experienced survey specialists. Then, they were back translated into English to ensure consistency. Data were collected by trained enumerators [17,21].

Our sample included 4727 mother–child dyads (15–49 years old) and (6–23 months old), respectively. The 2015/16 MDHS used the sampling frame for the 2008 Malawi Population and Housing Census. The survey employed a stratified two-stage probability sampling design in the country’s three main regions (northern, central, and southern) and formed a nationally representative sample. In the first stage, 850 clusters (173 in urban and 677 in rural areas) were selected; probability was proportional to the cluster size, and the selection was independent for each sampling stratum. In the second stage, 30 households per urban and 33 per rural cluster were selected using an equal probability systematic selection method. A detailed description of the survey methodology has been published elsewhere [17,22].

The article "Optimal Household Water Access Fosters the Attainment of Minimum Dietary Diversity among Children Aged 6–23 Months in Malawi" was retracted in 2021. Reasons: plagiarism; overlap with other authors' work.

### 2.2. Measurements

#### 2.2.1. Minimum Dietary Diversity

Our outcome variable was whether or not a child attained a minimally diverse diet assessed from data obtained through a simplified 24-h food questionnaire, which depended upon the mother’s ability to recall. The WHO defines a child as having attained MDD if the child was fed at least four of the following seven food groups during the previous 24 h: grains, roots, and tubers; legumes and nuts; dairy products (milk, yogurt, and cheese); flesh foods (meat, fish, poultry, and liver/organ meats); eggs; vitamin A rich fruits and vegetable; and other fruits and vegetables [3]. This was a binary variable which we coded as “1” if a child achieved MDD, and “0” if the child did not achieve MDD.

#### 2.2.2. Household Water Access

Household water access is a significant aspect of water insecurity and includes dimensions of sufficient quantity, as well as time spent on collecting water and meeting household needs [14,23]. We characterized water access levels based on an assessment of a household’s water sources. The DHS solicits information on household water sources through the question, “What is the main source of water used by your household for other purposes such as cooking and handwashing?” The response options include piped water, piped into dwelling, piped into yard/plot, bottled water, piped to neighbor, public tap, tube well water, tube well or borehole, protected well, protected spring, tanker truck, dug well, unprotected well, unprotected spring, river/dam, rainwater, and others.

Following the WHO standards [24], water access based on levels of needs met is defined as (1) basic or no access, when consumption needs are challenging to fulfill, and hygiene needs may or may not be assured; (2) intermediate, when consumption needs are assured and basic personal and food hygiene are met; and (3) optimal, when all consumption and hygiene needs are met.

From the MDHS data, we constructed our main predictor variable, i.e., household access to water, in the following manner:

1. Basic or no access, where water sources include dug well, unprotected well, unprotected spring, river/dam, rainwater, and others. In these cases, we expect that consumption needs may be met with difficulty, whereas minimum hygiene norms can hardly be assured.
2. Intermediate access, where water sources include piped to neighbor, public tap, tube well water, tube well or borehole, protected well, protected spring, and tanker truck. These sources are more likely to assure that consumption needs are met and that basic hygiene needs are likely to be met because even public sources are also protected.
3. Optimal access, where water sources include piped water, piped into dwelling, piped into the yard, and bottled water. We expect that among the available sources listed, these four sources are most likely to ensure water access in the desired quantity and quality, meeting all consumption and hygiene needs comfortably.

The article "Optimal Household Water Access Fosters the Attainment of Minimum Dietary Diversity among Children Aged 6–23 Months in Malawi" was retracted in 2021. Reasons: plagiarism; overlap with other authors' work.

This variable was constructed based on the WHO/United Nations Children’s Fund Joint Monitoring Program ladder for household water services [25], as well as Choudhary et al.’s coding system [26]. We excluded WASH-related variables from our analyses because the proposed pathways through which household water access affects dietary diversity are distinct from the WASH mechanism [26,27].

### 2.3. Covariates

We categorized our covariates into the following four levels: child, maternal, household, and community factors.

#### 2.3.1. Child Factors

Child factors included age (in months, 6–11, 12–17, or 18–23 months), sex (boy or girl), birth order (1, 2, 3, or 4+), and whether the child had diarrhea recently (yes or no).

#### 2.3.2. Maternal Factors

Maternal factors included age (in years, 15–24, 25–34, or 35–49), marital status (not married, married/cohabiting, divorced/separated/widowed), number of wives other than mother (0, 1, or 2+), educational level (no education, primary, secondary, or higher), occupation (housekeeping or agricultural, professional, service or manual labor), and breastfeeding duration (never breastfed, stopped breastfeeding, or still breastfeeding).

#### 2.3.3. Household Factors

Household (HH) factors included HH wealth index, number of HH members (1–5, 6–10, or 11+), number of children under 5 years (1, 2, or 3+), type of place of residence (urban or rural), and region (northern, central, or southern). The household wealth index was a composite measure of a household’s cumulative living standard and was derived according to a household’s ownership of selected assets, such as televisions and bicycles, materials used for constructing the house, access to safe water, sanitation facilities, and other household characteristics. Household asset scores were derived using a principal component analysis, thus, households were classified into quintiles (poorest, poorer, middle, richer, and richest) according to weighted household asset scores [28].

The article "Optimal Household Water Access Fosters the Attainment of Minimum Dietary Diversity among Children Aged 6–23 Months in Malawi" was retracted in 2021. Reasons: plagiarism; overlap with other authors' work.

#### 2.3.4. Community Factors

Community factors included the family planning method currently used (none, traditional/folkloric, or modern birth control), antenatal care attendance (ANC) during previous pregnancy (never attended, <4 visits (inadequate), or ≥4 visits (recommended)) [29], whether the mother received iron and folic acid (IFA) supplementation during the previous pregnancy (yes or no), whether the mother received malaria prophylaxis during the previous pregnancy (yes or no), and whether the mother received anthelminthic drugs during the previous pregnancy (yes or no).

### 2.4. Statistical Analysis

We performed all statistical analyses using SPSS Version 21.0 (IBM, Armonk, NY, USA) [30] and STATA version 14.1 (StataCorp, College Station, TX, USA) [31]. The STATA survey (svy) command was used to analyze the MDHS design effect. The participants’ characteristics were reported as weighted frequencies and percentages. Pearson’s Chi-square test was performed to assess the differences in the distribution of independent variables among groups (MDD, Yes/No) and check for possible confounding factors (Table S1). Variables with a *p*-value of < 0.05 were regarded as statistically significant. All significant independent variables in the univariable analysis were tested for multicollinearity using the variance inflation factor (VIF) [32,33] before being included in the final logistic regression analyses. One variable (marital status) was eliminated due to collinearity. No collinearity was observed among the rest of the independent variables, because all VIF values were <10 [34] (mean VIF 1.16).

Multivariable logistic regression analysis was performed by fitting the generalized estimating equation (GEE) to estimate the effects of the predictor variable on the outcome after all covariates were controlled for. The GEE model assumes a binomial distribution with a logit link function on the probability of parameters. Because of the MDHS data’s hierarchical structure, the GEE was used to adjust for any possible correlation in the responses of individuals (i.e., mother–child dyads) from the same clusters [35,36,37,38]. We applied a sampling weight in the GEE model. Additionally, we explored possible interaction effects among the covariates and household water access on MDD (Table S2). Crude and adjusted odds ratios (aORs) and their corresponding 95% confidence intervals (CIs) were derived. *K*-fold cross-validation was performed to estimate the accuracy of the predictive model in practice. The area under the curve was adequate to render the statistical analysis results generalizable to an independent dataset (Figure S1 and Table S3). The GEE-fitted multivariable analysis results were similar to those found using the generalized linear mixed model approach (Table S4).

The article "Optimal Household Water Access Fosters the Attainment of Minimum Dietary Diversity among Children Aged 6–23 Months in Malawi" was retracted in 2021. Reasons: plagiarism; overlap with other authors' work.

Subsequently, we performed a dominance analysis to determine the relative importance of the predictor variables relative to a child’s likelihood of achieving MDD; we estimated the explained variance using the McFadden R^2^ statistic [39]. Relative importance refers to an individual predictor variable’s proportionate contribution to R^2^ if we consider both its correlation with the outcome variable and its effect when combined with other predictor variables in the regression equation [40]. The general dominance weight for each predictor variable was divided by the combined general dominance weight of all predictor variables and multiplied by 100% to yield a normed measure representing each predictor’s proportion to the total variance. Dominance analysis accounts for an individual predictor variable’s direct effect, total effect (conditional on all other predictor variables), and partial effect (conditional on subsets of predictor variables) in terms of its contribution to the total variance [41,42,43].

### 2.5. Ethical Considerations

The 2010 and 2015/16 MDHSs were conducted according to the guidelines of the Declaration of Helsinki, and approved by the Institutional Review Board of ICF Macro, Maryland, USA, and the National Health Science Research Committee, Lilongwe, Malawi. Informed consent was obtained from all subjects involved in the study. The datasets are publicly available at http://dhsprogram.com/data/available-datasets.cfm upon approval of a written request.

## 3. Results

### 3.1. Sample Characteristics

Table 1 presents the characteristics of our study participants. Among the 4727 mother–child dyads (26.8 ± 6.8 years, range 15–49 years) and (13.9 ± 4.9 months, range 6–23 months), respectively, selected in this study, 27.7% of the infants and young children achieved MDD standards. This MDD prevalence is similar to that reported by the 2014 Malawi MDG Endline Survey [18]. The majority of the participants came from households with intermediate water access (79.5%), followed by households with basic or no water access (14.6%) and with optimal water access (5.9%). The children’s sex ratios were similar, and most children had no recent diarrheal disease.

Of the mothers, the majority were aged between 15 and 24 years (44.6%) and were either married or cohabiting (83.4%). Most mothers had only a primary-level education (67.1%) and were either homekeepers or engaged in subsistence farming (75.1%). Most of the mothers were still breastfeeding their children (88.5%) and came from households that (1) were classified as “poorest” (25.8%), (2) had between one and five members (57.5%), and (3) had only one child aged below five years (46.7%). Approximately half of the mothers had adequately attended the antenatal clinic during their previous pregnancy, most of whom received iron and folic acid supplementation (90.4%). Furthermore, 54.3% of the mothers were dewormed during their previous pregnancy.

The article "Optimal Household Water Access Fosters the Attainment of Minimum Dietary Diversity among Children Aged 6–23 Months in Malawi" was retracted in 2021. Reasons: plagiarism; overlap with other authors' work.

### 3.2. Minimum Dietary Diversity and Household Water Access

The Chi-squared measure of association between the percentage of children having achieved MDD and HH water access was statistically significant (*p* < 0.001, Table 2). Households with optimal water access had a higher proportion of children who achieved MDD than those with intermediate (58.4% vs. 26.6%) or basic/no water access (58.4% vs. 21.5%); the trend was similar for all the seven individual food groups (Figure 1). Another key finding was that complementary foods given to most children were mainly comprised of grains, roots and tubers and that dairy products and eggs were consumed infrequently (Figure 1).

### 3.3. Logistic Regression Results

Table 3 shows the predicted probability of a child’s achievement of MDD by household water access in Malawi. In the crude model, children had a higher probability of achieving MDD if they were from households with intermediate (OR = 1.32, 95% CI = 1.02–1.72) or optimal water access (OR = 5.16, CI = 3.49–7.62) as compared with children in households with basic or no water access. After adjusting for covariates, statistical significance persisted for households with optimal water access (aOR = 1.74, CI = 1.24–2.46). Children also had a higher probability of achieving MDD if they were older than 12 months, the odds increasing with age. In addition, children were more likely to achieve MDD if their mothers had a secondary-level education or higher (aOR = 1.61, CI = 1.21–2.13); had remunerated occupations (aOR = 1.26, CI = 1.08–1.48); and if they had been dewormed antenatally during their previous pregnancy (aOR = 1.18, CI = 1.04–1.35). Furthermore, compared with children from the poorest households, being from households with better financial status (poorer or higher) was positively associated with the achievement of MDD.

### 3.4. The Relative Importance of the Factors Associated with Minimum Dietary Diversity among Children Aged 6–23 Months, in Malawi

Table 4 reports the dominance analysis findings. In the model, household water access, a child’s age (in months), mother’s educational level, household wealth index, and type of area of residence were the top five variables among the nine evaluated. The top five variables accounted for 91% of the total variance (9%, 33%, 12%, 30%, and 7%, respectively).

The article "Optimal Household Water Access Fosters the Attainment of Minimum Dietary Diversity among Children Aged 6–23 Months in Malawi" was retracted in 2021. Reasons: plagiarism; overlap with other authors' work.

## 4. Discussion

Our results showed that only a small proportion (27.7%) of children achieved MDD, and it was positively associated with household water access among children aged 6–23 months, in Malawi. In addition, we found that infants and young children consumed complementary foods mainly comprised of grains, roots, and tubers. Similar dietary patterns were observed in Tanzania [44,45,46] and other sub-Saharan African countries [47,48]. Such dietary patterns may be attributable to water access as it affects household food diversity and food security through agricultural pathways. Agriculture is crucial for food security, more so in low-income countries such as Malawi [49]. However, food production requires access to substantial amounts of water; agriculture accounts for about 70 percent of the world’s water resources [50]. Despite water resources being abundant in Malawi, withdrawals remain very low; the total freshwater water withdrawals from developed water sources represents only 7.9 percent of total renewable water resources. This inadequacy in water development results from lack of financial, institutional, and technical means to invest in water infrastructure, and causes water to be a relatively scarce resource across the country [51]. Therefore, ninety percent of Malawi’s population largely depends on rain-fed agriculture to produce their food [52]. Unfortunately, rain-fed agriculture is directly exposed to the hazards of climate, resulting in unpredictable rainfall patterns. This renders large proportions of the population as food insecure on a yearly basis [52]. A report, by the Integrated Food Security Phase Classification, highlighted that between July and September 2020, about 10% of Malawi’s population faced high food insecurity due to floods and, subsequently, dry spells which led to shortfalls in agricultural production [53]. Access to sufficient amounts of water could potentially have averted this crisis. As a water-stressed country [20], most of Malawi’s rural population have lower opportunities to diversify their crops and produce a wider variety of foods due to insufficient water access. The literature has shown that people with greater access to water have better opportunities to diversify their crops than their counterparts in water-stressed regions [10].

Our findings also revealed that dairy products and eggs were consumed infrequently by young children. Limited opportunities to access these foods may be the main limiting factor for their regular consumption, as was observed in Tibet [54]. In addition to poor access, high cost may also inhibit their daily consumption among low-income families in Malawi. The finances for low-income families may further be strained by water access, as it may force them to choose between buying water, food, or fuel; purchasing water may render their finances insufficient for acquiring minimally diverse diets [7,12,13]. However, we found household water access to be an independent predictor of childhood dietary diversity even after adjusting for household financial status. Cultural beliefs and taboos may also undermine the consumption of the characteristic foods of Malawi. For instance, in some communities, there is a belief that eggs cause children to have abdominal pain, even develop epilepsy, and lead to baldness [55].

The article "Optimal Household Water Access Fosters the Attainment of Minimum Dietary Diversity among Children Aged 6–23 Months in Malawi" was retracted in 2021. Reasons: plagiarism; overlap with other authors' work.

Household access to water was ranked among the five most important predictors of children’s attainment of MDD in our dominance analysis, further highlighting the importance of the former on the latter. Our finding is consistent with that of Choudhary et al., who found that suboptimal household water access was associated with a lower probability of a child achieving MDD in India [26]. Household water access can also affect children’s attainment of MDD through gendered and competing demands on caregivers’ time [26]. The results from a 19-site cross-cultural study by Schuster and colleagues found that household water insecurity was qualitatively associated with children’s delayed feeding. Their mothers spent more time obtaining and managing water, and therefore compromised the time spent on food preparation to feed the children [15]. Our findings reinforced the existing literature that provided insights into the pathways through which household water access affected a child’s attainment of MDD [12,15,56]. Therefore, the present study may help to improve children’s dietary diversity, nutritional, and health outcomes. With the emerging trends in water access inequalities [20], strategies need to be put towards improving access to basic water services in the most vulnerable populations across all geographic and socioeconomic groups in Malawi in an effort to foster the achievement of MDD. Minimally diverse diets would provide infants and young children with vital macro- and micronutrients, thus, positively impacting their nutritional and health outcomes [26].

We also found that children older than 12 months of age had higher odds of meeting MDD than children aged 6–11 months. This finding is consistent with those of studies that were conducted in Tanzania [44], Ethiopia [57], Ghana [58], Sri Lanka [59], and India [60]. The finding implies that the practice of MDD increases as the child gets older. This might be due to poor exclusive breastfeeding, use of prelacteal liquids (e.g., herb teas), and late introduction of complimentary feeding [61,62]; when complimentary feeding is introduced on time, it mostly includes porridge made with white maize flour [63]. Another explanation could be that mothers perceive that a younger children’s digestive system might not cope with semi-solid and solid foods; some mothers fear that introducing bulk food would lead to infection [64]. Thus, education about complementary feeding should be geared towards mothers of younger children to encourage them to give children diversified diets with sufficient meal frequency. The 6–11-month age period coincides with the period with the highest risk of growth faltering [65]. Our result highlights the need to address suboptimal complementary feeding practices in this age group and to minimize growth faltering. Age, although not modifiable, represents a number of factors, especially the contextual environment and circumstances of a child’s rearing. It could well be that it embraces the broader family and maternal contributors to food and water quality.

The article "Optimal Household Water Access Fosters the Attainment of Minimum Dietary Diversity among Children Aged 6–23 Months in Malawi" was retracted in 2021. Reasons: plagiarism; overlap with other authors' work.

Furthermore, our study found that children whose mothers had attained at least a secondary-school-level education had a higher probability of achieving MDD. This finding is corroborated by studies from North West Ethiopia [66], Sri-Lanka [59], and five South Asian countries [67]. The studies showed that higher maternal educational level and overall literacy rate were significant determinants of infants’ and young children’s achievement of appropriate diversified feeding practices. The explanation for this could be that educated mothers are more likely to access higher quality health services and information. They might have learned about acceptable child feeding practices in their school curricula and were more likely to understand nutrition-education messages delivered through different media platforms quickly. Mothers with higher levels of education were more likely to be engaged in remunerative occupations and may, thus, be better off financially; this would afford their children a wider range of food items, therefore, increasing dietary diversity.

As compared with children whose mothers were either unemployed or depended on subsistence farming, children whose mothers were in remunerative occupations (i.e., professional/service/manual labor) were more likely to achieve minimum dietary diversity. This finding may be attributable to the fact that women with remunerative occupations may be in a better socioeconomic position to purchase sufficient amounts of foods required to achieve household food security, resulting in acceptable complementary feeding practices [68].

The article "Optimal Household Water Access Fosters the Attainment of Minimum Dietary Diversity among Children Aged 6–23 Months in Malawi" was retracted in 2021. Reasons: plagiarism; overlap with other authors' work.

Using household wealth index as a proxy for household socioeconomic status, the present study exhibited an upward trend in children’s achievement of MDD with increasing wealth quintiles, indicating a relationship between household wealth and feeding practices. This finding is supported by those from Nepalese [69] and Ethiopian [70,71] studies. A possible explanation for this finding is that parents from wealthier households are more likely to access and afford more diverse foods to feed their children than their counterparts from low-income households. Our dominance analysis ranked the household wealth index as the most important modifiable factor associated with a child’s attainment of MDD among the ten variables analyzed. This finding underscores the need to strengthen interventions that promote food accessibility for low-income households, including the promotion of husbandry practices and the use of the resulting food products [34]. Hence, we recommend enhancing programs that integrate interventions geared toward improving maternal education, food accessibility, and overall household socio-economic status in Malawi.

This study found that households with two children under five years of age were less likely to provide the children with minimally diverse diets. Other than in multiple gestations, having more than one under-five-year-old child may signify that a woman has frequent and high parity. Tegegne et al. reported increased odds of appropriate child-feeding practices among mothers with low parity in Ethiopia [72]. Therefore, the explanation for our finding could be that having more than one child under five years of age reduces a mother’s level of attention for her children, which may influence a lower level of childcare, commitment, and motivation to follow appropriate child-feeding practices.

Finally, children whose mothers received anthelmintic drugs during their last pregnancy were more likely to achieve MDD. The explanation for this may be that mothers’ knowledge about complementary feeding practices improved with exposure to health professionals after receiving counseling from the health practitioners during their antenatal care visits. Similar observations and assertions were made by Iqbal et al. [73] and Joshi et al. [69] in their Bangladeshi and Nepalese studies, respectively.

## 5. Strengths and Limitations

The present study applies dominance analysis to regression models to ascertain the association and relative importance of household access to water in Malawian children’s attainment of MDD. Our findings have offered insights and generated hypotheses regarding policy, societal, and household factors, which might account for associations found previously and elsewhere but requiring confirmation in Malawi. This study utilized a large sample size which employed high-quality control measures and used contextual variables in child, maternal, household, and community-level adjustments. Thus, a clearer picture of the role that household access to water plays on the achievement of MDD among infants and young children in Malawi has been possible.

The article "Optimal Household Water Access Fosters the Attainment of Minimum Dietary Diversity among Children Aged 6–23 Months in Malawi" was retracted in 2021. Reasons: plagiarism; overlap with other authors' work.

Interpretation of our findings is limited by the cross-sectional nature of the data, which only allows correlative rather than causative conclusions. Nonetheless, our results unravel possible pathways linking water to MDD, which can be explored further using other analytical approaches. Moreover, the study utilized secondary datasets, which, although large, lacked variables which could have resolved some outstanding questions. For instance, as was the case with Choudhary et al.’s study [26], our data lacked variables for assessing a caregiver’s time allocation across the management of household water resources or childcare activities and how water access affected cooking patterns and irrigation activities, which restricted us from gaining a deeper understanding of the underlying associations. Since access to clean water is part of the household wealth index, collinearity may impair the deduction that water accessibility accounts for MDD. However, from the VIF (1.16) and the sensitivity analysis with and without the household wealth index (Table S5), no severe violation of the validity of the model was found. A thoroughly contextual approach to our hypothesis is necessary requiring a range of covariates. These have been chosen as those of most likely import, although residual confounding is inevitable. In addition, the attainment of MDD among infants and young children was assessed using a binary variable that might have attenuated some precision in measuring the data. Lastly, the DHS data were based on a questionnaire and prone to fallible memory.

## 6. Policy Implications

The findings of our analysis build on the existing literature that provides insights into how household water access might affect a child’s attainment of MDD. Therefore, incorporating water-based strategies into national nutrition policies may help to improve childhood dietary diversity and reduce the burden of childhood undernutrition in Malawi.

## 7. Conclusions

Our study builds on the emerging body of evidence that suboptimal access to water resources provides additional pathways to child nutrition through access to, and availability of minimally diverse diets. Developing strategies for increasing access to water may positively impact child nutritional status, especially in resource-constrained households.

The article "Optimal Household Water Access Fosters the Attainment of Minimum Dietary Diversity among Children Aged 6–23 Months in Malawi" was retracted in 2021. Reasons: plagiarism; overlap with other authors' work.

## Figures and Tables

**Figure 1:** Infants’ and young children’s food consumption proportions per food group relative to household water access.

**Table 1:** Sociodemographic characteristics of the study participants (*n* = 4727).

Characteristics	Proportion
	*n* (%)
Infant and child minimum dietary diversity, Achieved	1311 (27.7)
Household Water Access	
Basic or no access	689 (14.6)
Intermediate	3759 (79.5)
Optimal	279 (5.9)
Child Factors	
Child’s age (months), mean (SD)	13.9 (4.9)
6–11	1618 (34.2)
12–17	1636 (34.6)
18–23	1473 (31.2)
Sex, girl	2310 (48.9)
Child had diarrhea recently, Yes ^††^	1845 (39.1)
Maternal Factors	
Mother’s age (years), mean (SD)	26.8 (6.8)
15–24	2108 (44.6)
25–34	1886 (33.9)
35–49	732 (15.5)
Marital status	
Not married	223 (4.7)
Married/cohabiting	3944 (83.4)
Divorced/separated/widowed	560 (11.9)
Mother’s educational level	
No education	563 (11.9)
Primary	3172 (67.1)
Secondary or higher	992 (21.0)
Occupation	
Housekeeping/agriculture	3552 (75.1)
Professional/service/manual labor	1174 (24.9)
Breastfeeding duration ^††^	
Never breastfed	48 (1.0)
Stopped breastfeeding	495 (10.5)
Still breastfeeding	4184 (88.5)
Household Factors	
Household wealth index	
Poorest	1218 (25.8)
Poorer	1080 (22.8)
Middle	912 (19.3)
Richer	7876 (16.6)
Richest	731 (15.5)
Number of children under the age of 5 years ^††^	
1	2195 (46.7)
2	2124 (45.1)
3+	385 (8.2)
Type of area of residence, Rural	4086 (86.4)
Community Factors (Community Health Services)	
Family planning method currently used	
None	1446 (30.6)
Traditional/folkloric	47 (1.0)
Modern birth control	3234 (68.4)
Received anthelmintic drugs during the previous pregnancy, Yes	2561 (54.3)

^††^ Total count is less than *N*; HH, household; IFA, iron and folic acid; SD, standard deviation.

**Table 2:** Proportion (in %) of infants and young children aged 6–23 months achieving minimum dietary diversity by household water access in Malawi (*n* = 4727).

Characteristics	Minimum Dietary Diversity		*p*
	No	Yes	
	*n* (%)	*n* (%)	
Household Water Access			<0.001
Basic or no access	541 (78.5)	148 (21.5)	
Intermediate	2759 (73.4)	1000 (26.6)	
Optimal	116 (41.6)	163 (58.4)	

*p*, Pearson’s Chi-square *p*-value. Statistical significance was set at *p* < 0.05.

**Table 3:** Association between household water access and minimum dietary diversity among children aged 6–23 months in Malawi. Crude and adjusted odds ratios based on generalized estimating equation (GEE)-fitted logistic regression analysis (*n* = 4727).

Characteristics	Minimum Dietary Diversity	
	OR (95% CI)	aOR (95% CI)
Household Water Access		
Basic or no access	1.00 (ref)	1.00 (ref)
Intermediate	1.32 (1.02–1.72)	1.08 (0.87–1.35)
Optimal	5.16 (3.49–7.62)	1.74 (1.24–2.46)
Child Factors		
Child’s age (months)		
6–11	1.00 (ref)	1.00 (ref)
12–17	2.27 (1.82–2.83)	2.26 (1.89–2.69)
18–23	2.82 (2.28–3.48)	2.79 (2.35–3.31)
Maternal Factors		
Mother’s educational level		
No education	1.00 (ref)	1.00 (ref)
Primary	1.76 (1.32–2.34)	1.19 (0.93–1.53)
Secondary or higher	3.39 (2.46–4.69)	1.61 (1.21–2.13)
Occupation		
Housekeeping/agriculture	1.00 (ref)	1.00 (ref)
Professional/service/manual labor	1.86 (1.53–2.24)	1.26 (1.08–1.48)
Household Factors		
Household wealth index		
Poorest	1.00 (ref)	1.00 (ref)
Poorer	1.54 (1.18–2.02)	1.36 (1.10–1.68)
Middle	1.90 (1.46–2.47)	1.55 (1.26–1.92)
Richer	2.44 (1.85–3.22)	1.97 (1.56–2.48)
Richest	4.78 (3.57–6.42)	2.64 (2.00–3.48)
Number of children under the age of 5 years		
1	1.00 (ref)	1.00 (ref)
2	0.68 (0.57–0.81)	0.84 (0.73–0.97)
3+	0.83 (0.67–0.99)	1.05 (0.82–1.36)
Type of area of residence		
Rural	1.00 (ref)	1.00 (ref)
Urban	0.36 (0.28–0.46)	1.06 (0.83–1.34)
Community Factors (Community Health Services)		
Family planning method currently on		
None	1.00 (ref)	1.00 (ref)
Traditional/folkloric	2.71 (1.20–6.09)	1.64 (0.90–3.00)
Modern birth control	1.35 (1.13–1.61)	1.04 (0.91–1.20)
Received anthelmintic drugs during the previous pregnancy		
No	1.00 (ref)	1.00 (ref)
Yes	1.22 (1.06–1.41)	1.18 (1.04–1.35)

OR, odds ratio; aOR, adjusted odds ratio; CI, confidence interval; GEE, generalized estimating equation. Statistical significance was set at *p* < 0.05.

The article "Optimal Household Water Access Fosters the Attainment of Minimum Dietary Diversity among Children Aged 6–23 Months in Malawi" was retracted in 2021. Reasons: plagiarism; overlap with other authors' work.

**Table 4:** Dominance analysis to determine the relative importance of the factors associated with minimum dietary diversity among children aged 6–23 months, in Malawi (*n* = 4727).

Variables	Minimum Dietary Diversity		
	Dominance Statistic	Standardized Weight ^††^	Rank
Household water access	0.0074	0.09	4
Child’s age (months)	0.0269	0.33	1
Mother’s educational level	0.0099	0.12	3
Occupation	0.0050	0.06	6
Household wealth index	0.0240	0.30	2
Number of children under the age of 5 years	0.0010	0.01	7
Type of area of residence	0.0053	0.07	5
Family planning method currently used	0.0003	0.01	9
Received anthelmintic drugs during the previous pregnancy	0.0010	0.01	8
Overall fit statistic	0.0808		

^††^ Standardized weight is the general dominance weight from McFadden R^2^ normed or standardized to be out of 100%. Variables included in this dominance analysis are those fitted into the final regression model.

## Supplementary Materials

The following are available online at https://www.mdpi.com/2072-6643/13/1/178/s1, Figure S1: A graphical illustration of the *K*-fold cross-validated ROC curve for estimating the accuracy of the predictive model for testing the association between household water access and MDD among 6–23 month-old children in Malawi, Table S1: Chi-squared associations between demographic characteristics and MDD (*n* = 4727), Table S2: Interactions of household water access with other independent variables in predicting the achievement of minimum dietary diversity (*n* = 4727), Table S3: *K*-fold cross-validation for estimating the accuracy of the predictive model for testing the association between household water access and minimum dietary diversity among 6–23 month-old children in Malawi (*n* = 4727), Table S4: Association between household water access and minimum dietary diversity among children aged 6–23 months in Malawi: crude and adjusted odds ratios based on GLMM-fitted logistic regression analysis (*n* = 4727), Table S5: Association between household water access and minimum dietary diversity among children aged 6–23 months, in Malawi: crude and adjusted odds ratios based on GEE-fitted logistic regression analysis (with and without household wealth index) (*n* = 4727).
